# Effect of the Specific Training Course for Competency in Doing Arterial Blood Gas Sampling in the Intensive Care Unit: Developing a Standardized Learning Curve according to the Procedure's Time and Socioprofessional Predictors

**DOI:** 10.1155/2021/2989213

**Published:** 2021-02-13

**Authors:** Amir Vahedian-Azimi, Farshid Rahimi-Bashar, Mohamad-Amin Pourhoseingholi, Mahmood Salesi, Morteza Shamsizadeh, Tannaz Jamialahmadi, Keivan Gohari-Moghadam, Amirhossein Sahebkar

**Affiliations:** ^1^Trauma Research Center, Nursing Faculty, Baqiyatallah University of Medical Sciences, Tehran, Iran; ^2^Department of Anesthesiology and Critical Care, School of Medicine, Hamadan University of Medical Sciences, Hamadan, Iran; ^3^Department of Health System Research, Research Institute for Gastroenterology and Liver Diseases, Shahid Beheshti University of Medical Sciences, Tehran, Iran; ^4^Chemical Injuries Research Center, Systems Biology and Poisonings Institute, Baqiyatallah University of Medical Sciences, Tehran, Iran; ^5^Chronic Diseases (Home Care) Research Center, Hamadan University of Medical Sciences, Hamadan, Iran; ^6^Department of Food Science and Technology, Quchan Branch, Islamic Azad University, Quchan, Iran; ^7^Department of Nutrition, Faculty of Medicine, Mashhad University of Medical Sciences, Mashhad, Iran; ^8^Medical ICU and Pulmonary Unit, Shariati Hospital, Tehran University of Medical Sciences, Tehran, Iran; ^9^Biotechnology Research Center, Pharmaceutical Technology Institute, Mashhad University of Medical Sciences, Mashhad, Iran; ^10^Applied Biomedical Research Center, Mashhad University of Medical Sciences, Mashhad, Iran; ^11^School of Pharmacy, Mashhad University of Medical Sciences, Mashhad, Iran

## Abstract

**Background:**

Standardization of clinical practices is an essential part of continuing education of newly registered nurses in the intensive care unit (ICU). The development of educational standards based on evidence can help improve the quality of educational programs and ultimately clinical skills and practices.

**Objectives:**

The objectives of the study were to develop a standardized learning curve of arterial blood gas (ABG) sampling competency, to design a checklist for the assessment of competency, to assess the relative importance of predictors and learning patterns of competency, and to determine how many times it is essential to reach a specific level of ABG sampling competency according to the learning curve.

**Design:**

A quasi-experimental, nonrandomized, single-group trial with time series design. *Participants*. All newly registered nurses in the ICU of a teaching hospital of Tehran University of Medical Sciences were selected from July 2016 to April 2018. Altogether, 65 nurses participated in the study; however, at the end, only nine nurses had dropped out due to shift displacement.

**Methods:**

At first, the primary checklist was prepared to assess the nurses' ABG sampling practices and it was finalized after three sessions of the expert panel. The checklist had three domains, including presampling, during sampling, and postsampling of ABG competency. Then, 56 nurses practiced ABG sampling step by step under the supervision of three observers who controlled the processes and they filled the checklists. The endpoint was considered reaching a 95 score on the learning curve. The Poisson regression model was used in order to verify the effective factors of ABG sampling competency. The importance of variables in the prediction of practice scores had been calculated in a linear regression of R software by using the relaimpo package.

**Results:**

According to the results, in order to reach a skill level of 55, 65, 75, 85, and 95, nurses, respectively, would need average ABG practice times of 6, 6, 7, 7, and 7. In the linear regression model, demographic variables predict 47.65 percent of changes related to scores in practices but the extent of prediction of these variables totally decreased till 7 practice times, and in each practice, nurses who had the higher primary skill levels gained 1 to 2 skill scores more than those with low primary skills.

**Conclusions:**

Utilization of the learning curve could be helpful in the standardization of clinical practices in nursing training and optimization of the frequency of skills training, thus improving the training quality in this field. This trial is registered with NCT02830971.

## 1. Introduction

Standardization of clinical practices is an essential component of nursing education; nursing education is an expensive and time-consuming task, and other problems like the heavy load of the nursing educator's work and lack of human resources and facilities of standard education complicate the educational process [1]. Nursing education is a practical field, and to develop skills, one needs to learn theoretical knowledge and clinical practice simultaneously in the educational environment; due to the importance of primary skills of nurses in their subsequent competency and the significant role of nurses in any stage of the procedure, it is better to recruit empowered nurses with higher primary competencies especially in the intensive care unit (ICU) [2, 3]; ICU is a critical unit, and most critically ill patients are admitted to it, so any medical error can threaten the patient's life; therefore, it is necessary to standardize nursing practice times of any skills according to updated learning process models.

The learning process consists of studying knowledge and frequently practicing the skills to achieve clinical competence [4]. Clinical competency means the ability to perform actions with the standards of the nursing profession, which have multidimensional nature and involve technical, cognitive, and emotional abilities [5].

According to Benner's theory, the repetition of skills leads to gradual skill development [6]. The evidence showed that increasing the frequency of clinical skills would lead to the development of the nurse's competency [7], but the number of times required to develop the maximum individual competency in any special clinical skill is currently being studied.

Previous studies have shown that newly registered nurses do not experience all skills equally. Some skills like measurement of blood pressure and body temperature are performed repeatedly, but skills like monitoring a chest tube and endotracheal tube are experienced by only a few [8].

Sampling of arterial blood gas (ABG) by the direct vascular puncture is an invasive procedure often practiced in ICU settings. Since ABG is invasive and done in critically ill patients, it is an important learning issue in nurse training, and newly registered nurses must be competent in ABG sampling during their training courses in the ICU [9].

Achievement of clinical competency and its determination are critical issues in nursing education. It can be assessed by checking technical, cognitive, and emotional abilities in any experience, and the process of skill conducting is continued until it is done in the standard criteria [10]. This method is called the “learning curve” and shows the development of individual skills in the repeated experiences.

The learning curve was used for the first time in psychology to represent the relationship between practice and related changes in behavior [11]. Previously, in medical education, this method was used to evaluate the different learning practices [12, 13]. The concept of the plateau in the learning curve has not been certified and accepted everywhere as a standard level of learning [14].

The learning curve is a diagram showing the increase of learning (vertical axis) with multiexperiences (horizontal axis) [15]. It has been used to describe improvements in human performance in a wide range of domains [16–18]; in most studies, “the learning curve reaching the plateau” is considered to be the criteria for achieving competency [19]. The plateau level may change a little, but changing a little in the plateau level means important further progress in proficiency.

In the nursing field, no definitive standard of the frequency of any practices has been defined for competency achievement yet, which may be because of the multidimensional nature of practice education in the clinical field [20].

Considering the rapid progress of training techniques, it seems nursing education should be updated and efficient; furthermore, the development of educational standards based on evidence can help improve the quality of educational programs for newly registered working nurses in the ICU.

### 1.1. Study Purpose

The purpose of the study was fourfold:

1. Designing a checklist for the assessment of nurses' ABG sampling competency
2. Determining how many times it is essential to reach a specific level of ABG sampling competency according to the learning curve
3. Assessing the relative importance of predictors and learning patterns of ABG sampling competency
4. Developing a standardized learning curve for ABG sampling competency

## 2. Method

### 2.1. Study Design

This study is a quasi-experimental, nonrandomized, single-group trial with time series design in three phases of the study.

### 2.2. Samples and Setting

All newly registered nurses in the ICU from July 2016 to April 2018 were selected for the study through convenience and sequential samplings to fulfill the inclusion criteria in the teaching hospital affiliated with Tehran University of Medical Sciences (TUMS). The prolonged selection sample was related to less displacement of ICU nurses and changing the working nurses there; moreover, there were fewer newly registered nurses in the ICU, hence less displacement of ICU working nurses. The ICU had 10 mixed beds, which were for hospitalized medical and surgical patients, with 28 working nurses totally. The turnover rate of the patients was twelve to fifteen surgical patients and three to eight medical patients each week.

The sample size was determined based on the power assumption of 90% and the significance level of 0.05. The method of convenience and sequential sampling was developed, so the times of sample selection and interventional period were simultaneous, and the study lasted about 22 months. During the study period, 65 nurses who were recruited from the newly registered nurses participated in the study. They passed the skill course according to the curriculum in the ICU before entering the study. At the end, 56 nurses remained and 9 nurses had dropped out due to changing to ward duty in the study period.

### 2.3. Data Collection

As the first phase of the study, a checklist was created for data collection (Figure 1) according to three expert panel sessions. In the first step, an extensive review of the literature was done based on the latest documents and articles in the procedure of ABG sampling, including 23 original papers, 8 review papers, and 5 nursing textbooks. The members of the expert panel (*n* = 28) were three intensivists, five anesthesiologists, three pulmonologists, five internists, a nephrologist, a cardiologist, and ten highly experienced ICU nurses (the nurses who have worked for more than 20 years in ICU settings). Kendall's agreement coefficient of the expert panel for selecting primary materials for constituting the checklist was 0.976 (*P* value < 0.0001). The primary checklist was prepared, and it was introduced in the first expert panel. Primary consensus about the checklist was achieved after a 90-minute discussion. Then, the primary checklist was sent to expert members for polishing, improving, and editing. The results of the second session (lasting 120 min) were analyzed meticulously by the principal investigator and two independent researchers (*K* = 0.943 with *P* value < 0.0001). Then, the third version of the checklist was prepared based on the results of the second session, and finally, the main checklist of the clinical survey was prepared according to the last session (lasting 120 min).

During the three validation sessions, the content validity ratio was 0.59 (CVR = 0.59) and the content validity index was 0.95 (CVI = 0.95) with 28 panelists. Reliability of the checklist was determined based on the interrate reliability with the Kappa agreement test by the principal investigator with intensivists (*r* = 0.94), anesthesiologists (*r* = 0.92), pulmonologists (*r* = 0.90), internists (*r* = 0.93), nephrologists (*r* = 0.97), a cardiologist (*r* = 0.95), and three of the nurses (*r* = 0.91, 90, and 92) separately. Reliability of the checklist was determined based on the intrarate reliability with the Kappa agreement test by the principal investigator (*r* = 0.96), intensivists (*r* = 0.91), anesthesiologists (*r* = 0.92), pulmonologists (*r* = 0.94), internists (*r* = 0.92), nephrologists (*r* = 0.93), a cardiologist (*r* = 0.90), and three of the nurses (*r* = 0.90, 93, and 94) separately.

Other variables of the study that were included were GPA (Graduate Point Average), gender, age, preeducation status, shift work, cooperation, major satisfaction, and supervisor.

### 2.4. Intervention

The second phase of our study included intervention and data collection (Figure 1). During the intervention, three observers from the ICU staff controlled the ABG sampling processes of each nurse every time (in each shift when the newly registered nurses wanted to get the ABG sample) and they filled the checklists.

All participants were newly graduated and registered as an ICU nurse. The nurses were taught theoretical and practical skills of ABG sampling previously during their studentship period. Doing the procedure was the first time for the participants. Nurses received full education according to the final checklist components by a full-time ICU trainer in five 120 min sessions theoretically; although the trainers were informed about the general method of research, they were not told about the research questions. Three observers from the highly experienced ICU staff were trained to fill the checklists during the study. The endpoint was considered reaching a 95 score on the learning curve. The reason for selecting less than 5 percent variation is because of being equal to the flattening of the learning curve (the plateau section) [21]. Inclusion criteria included consent to participate in the study, had not already done the technique in the ICU, passing prerequisite courses, and not having any problem doing ABG sampling. The results of the two primary weeks were not considered (for each participant) to decrease the researcher effects on the participants. Following each newly registered nurse was continued until the flattening of the learning curve was reported.

### 2.5. Ethical Considerations

The present study was registered with the research committee of the hospital, and the research package was explained clearly to hospital authorities. The ethical considerations were related to the nurses' autonomy, confidentiality, and anonymity during the study period and its publication. The objectives of the study were explained to all nurses, and they were also informed they were free to participate, decline participation, or withdraw from the study any time they pleased. Written informed consent was obtained from the nurses who agreed to be included in the study.

### 2.6. Data Analysis

In the study, the Poisson regression model was used in order to verify the effective factors on the frequency of practices to reach a specific level of ABG competency. Nine Poisson models were fit to the data according to the necessary practice times to reach the skill scores, including 55, 60, 65, 70, 75, 80, 85, 90, and 95 with predictable variables of GPA, gender, age, preeducation score, shift, cooperation, and supervisor. For each model (each cutoff point), the predicted values of the model (aligned) were evaluated in contrast with the main values, and according to the following calculation, the accuracy of the model was gained in the estimation of the necessary practice times to reach a specific level of competency. Finally, the best Poisson model was reported with the best accuracy for prediction and identification and best results [22].

(1) $$\begin{array}{c} \text{Accuracy percentage}=\frac{\left(\#\text{actual times}=\text{rounded predicted times}\right)}{\text{sample size}}\times 100. \end{array}$$

The average of the necessary practice times to reach each cutoff point with its distribution, the box plot, and the average of learning levels were reported in two groups with high and low primary skill levels via a learning curve diagram in 7 practices. The nurse's skills were categorized according to the average of the primary skills (those who were less than the average were labeled as low, and others were supposed to be high or on normal level). Also, the relative importance of the mentioned demographic variables in the prediction of practice scores had been calculated in a linear regression of R software by using the relaimpo package. The relative importance was actually the resolution of *R*^2^ for the linear regression model, specifying the proportion of each variable from the total predicted changes in a way that the sum of each of these effects was equal to *R*^2^ of the model. The greater the value demonstrated, the greater the importance and the more impact the variables have on the linear model. All analyses were done using the R software and the relaimpo package.

## 3. Results

### 3.1. Description of Participants

Fifty-six nurses participated in the study, including 19 (33.9%) males and 37 (66.1%) females. The total mean age of participants was 24.6 (±1.5 SD) years; it was 24.2 (±1.9 SD) years in men and 24.8 (±1.3 SD) years in women separately. There was no significant difference in the mean age of men and women. The mean GPA of participants was 16.9 (±1.4 SD) from 20, and it was not significantly different in men and women (Table 1).

### 3.2. Designing the Checklist

The final checklist had three domains, including pre-ABG sampling (5 questions), during ABG sampling (8 questions), and post-ABG sampling (5 questions). The scoring of each question was based on the 3 statuses of the following: ability to perform alone (score 2), ability to perform with help (score 1), and inability to perform (score 0). Each question had a specific importance coefficient among 1 to 5. The philosophy of different coefficients of questions in three domains was related to the importance degree of the question. Thus, besides the domain scores, each domain had a specific importance coefficient. The total score of the checklist comes from multiplying the question score to the question importance coefficient in percentage. Thus, the highest score of the checklist was 100 percent and the lowest was 0 percent (Table 2).

### 3.3. Essential Times to Reach a Specific Level according to the Learning Curve

#### 3.3.1. Skill Scores in Different Practices for ABG Sampling Competency

Figure 2 (the box plot of skill scores across different practice frequencies) shows that, in each repetition of practices, it ended at the higher level of scores, including 30 as the first practice score, and it ended higher than 95 at the last practice repetition (7th). When repeating the practice, the nurse's skill scores increased on average 10 points (Figure 2). The maximum gained score of competency in the 1st to 7th practices was, respectively, 40, 54, 64, 77, 89, 99, and 100. By increasing the practice time, the variation of skill scores increased and the range of scores in each practice time was totally different. Most fluctuation and dispersion of skill scores among nurses were in the 4th and 6th practices.

#### 3.3.2. Frequency of Steps to Reach a Specific Level of Skill for ABG Sampling Competency

Figure 3 indicates the ABG skill scores in two groups of high and low primary skill levels. The growth rate of both was almost equal and increased in a parallel manner. This figure shows that the nurses, who had higher primary skill levels, were expected to have higher skill levels mainly in later practices; in other words, in each practice, nurses who had the higher primary skill levels gained 1 to 2 points more than nurses with low primary skills. This illustrated that the frequency of steps to reach a specific level of skill is relatively dependent upon the basic level of proficiency. However, both groups reached 75% of skills after 5 practices.

#### 3.3.3. Increasing Skill Scores in Each Practice for ABG Sampling Competency

The extent of increasing skill scores for each practice time, compared to the previous step, is shown in Figure 4. The impact of practices on increasing the competency decreased from the first to the third steps. Then, in the 4th and 5th steps, an increase was observed in the mentioned values. The greatest increase was observed in the first and fifth steps, compared to the subsequent and previous steps. Ultimately, in the two latest steps, the rate of increase was decreased in a way that it reached the least value in the last step. In other words, the changing of competency values was not in a linear trend and mostly appeared in a sinusoidal shape (first decreasing, then increasing, and decreasing again after that).

#### 3.3.4. Predicted Time Accuracy for ABG Sampling Competency

Figure 5 presents the average necessary times to reach the different levels of ABG proficiency, which were reported in 7 measurement times for each nurse by the dashed line. According to the results, in order to reach the skill level of 55, 65, 75, 85, and 95, nurses would need an average ABG practice time of 6, 6, 7, 7, and 7, respectively. In other words, with 5 practice times, nurses would reach the competency score of 55, with 6 practice times, they will reach the score of 75, and with 7 practice times, they would have a remarkable increase to the competency score of 95.

#### 3.3.5. Necessary Times to Reach the ABG Sampling Competency by the Segregation of Nurses

Figure 6 shows the scatter of necessary times to reach the different levels of competency by the segregation of nurses. According to this figure, to reach the scores of 75 to 85, 4 practice times were needed for 8 nurses, and to reach a score of 90, 5 practice times were needed for 2 nurses that had better conditions in contrast to the average of nurses.

#### 3.3.6. Relative Importance of Predictors in ABG Sampling Competency

Multiple linear regression analysis indicated that demographic variables predicted 47.65 percent of changes in the related score in practices. But the extent of prediction of these variables totally decreased to 7 practice times, as it decreased to 24.35 percent of total changes, which means that the predictability decreased almost half of its percentage in the first practice (Table 3). The major satisfaction variable had shown a significant impact on the related score till the 5th practice (except the 4th ones), but it was not effective in more practices. While the impact of the preeducation variable decreased as the number of practices increased and after the 5th practice, it had nonsignificant effects on skill scores. The greatest impact of this variable was in the first and second practice times. Although the rest of the variables in each of the practice times did not show any significant association, considering the relative importance of sex and colleagues' cooperation variables, a declining rate of the importance in increasing the steps was shown, and in other variables, they had a fixed rate or did not show a specific rate.

#### 3.3.7. Developing a Standardized Learning Curve for ABG Sampling Competency

In Poisson models, which are designed for verification of the effect of different factors on necessary times to reach the different levels of learning, all of the variables had the potential predictability by the Poisson regression model simultaneously as 25, 37.5, 64.3, 80.4, and 96.4 percent of nurses in fulfilling the necessary practice times to reach the skill level of 55, 65, 75, 85, and 95. These results implied that the designed Poisson models with the mentioned variables can predict the necessary practice times to reach the skill level of 75 to 95 with good accuracy. But to reach a score of less than 70, it could not be helpful, and the accuracy of the Poisson model would be less than 50 percent (Figure 7).

## 4. Discussion

This study was one of the first studies in the field of nursing education, which was conducted based on the learning curve for competency in doing arterial blood gas sampling in the ICU and which developed a standardized learning curve based on the procedure's time and socioprofessional predictors.

In this study, the extent of the nurse's competency in repeated times of ABG sampling was determined and it was registered in the learning curve. Results show that in order to reach the skill level of 55, 65, 75, 85, and 95, nurses, respectively, nurses would need average ABG practice times of 6, 6, 7, 7, and 7. This means that the nurses would reach the competency score of 95 by practicing 7 times. The greatest increase of ABG sampling competency due to practicing was observed in the first and fifth steps in comparison to the subsequent and previous steps. In the linear regression model, demographic variables predict 47.65 percent of changes in the related score in practices, but the extent of prediction of these variables totally decreased until 7 practices had been done. Major satisfaction showed a meaningful impact on the related score until the 5th practice, and the impact of the preeducation variable decreased by increasing the practice until the 5th practice. Gender and colleagues' cooperation variables showed a declining rate of importance in increasing the practice steps. The related variables in Poisson models can predict the necessary practice times to reach a skill level of 75 to 95 with almost good accuracy. But to reach a score before 70, it could not be helpful, and the accuracy of the Poisson model would be just under 50 percent.

Arterial blood gases are judicable only if obtained properly and analyzed accurately. Some studies determined that some preanalyzed factors affected the validity of ABG sampling results and may be due to adverse patient management [23]. So, in the first step, the checklist was designed for this study in three stages: before (included 5 items), during (included 8 items), and after (included 5 items) the procedure. The development and validation method of a checklist to assess ABG sampling competency may be critical because the well-defined structure of the checklist sequenced coherent practices and measurements and reliable results in which it is to be applied.

Considering the items of checklists such as syringe preparation, patient handling, and sample controlling, the nurse's role is very important due to the production of accurate results; moreover, this study showed that nurses who had a high level of primary skills have obtained a higher score in contrast to people with prior lower skills. As a result, the expected experience times to reach a special level of competency in a relative mode depend on the basic skill level.

Grantcharov et al. also considered the needed times for acquiring competency in laparoscopy depending on the prior proficiency of physicians. The first level of proficiency reached a plateau level of the learning curve after 2 repetitions, while the second level of proficiency reached a plateau after repeating 5 times and the third level of proficiency reached a plateau after repeating 7 times [24]. In Loukas et al.'s study, the learning curve of novices in IV cannulation reached a plateau level after 8 times, while in intermediates, it reached a plateau level after 6 times [25]. This flexibility is an advantage of the learning curve method, which can be used to predict the expected frequency for obtaining competency in any level of primary skills of participants.

Results showed an increasing rate of skill scores in each practice, especially in the first five steps. Park et al. also showed that with an increase in the times of doing the laparoscopic resection surgery of colorectal cancer, participants' competence increased and surgery duration and its side effects reduced, particularly in the early stages [26]. This result shows the importance of the first steps of training of nurses and its impact in enhancing their ability, so it may be necessary to supervise the nurses during the first time of their accurate practicing.

The maximum scores of skills were 40, 54, 64, 77, 89, 99, and 100 from the 1st to 7th steps, respectively. This score may be helpful in developing an educational curriculum and designing courses for nurse training. The practice times of other skills were standardized with this method previously. But no studies have been done in the case of ABG sampling competency learning.

In Loukas et al.'s study, in the case of IV cannulation, the learning curve reached a plateau level after 6 times of experience [25]. Grantcharov et al. mentioned that 2 to 7 practice times may be needed to become proficient in cystoscopy [24].

Thomas believed that it is better to utilize this method in proficiency, which has complex cognitive and psychological levels of learning [27]. Regarding the multidimensional concept of nursing education, utilization of the learning curve would be proper in this field. Furthermore, although the competency level may rise after flattening the learning curve with replication of skills, the rate of increase in contrast to the costs and other consequences may be very little and the nurses may have the opportunities to acquire this progress at later stages of clinical tasks.

This study indicated that demographic variables predict 47% of changes in skill scores. According to prior studies, proficiency type, acting stages, and personal characteristics could be effective in the extent of acquiring competency [28]. Other studies implied that demographic factors like gender and ethnicity would be significant predictors of success in medical education. But they did not mention the extent of prediction [29, 30]. Considering these factors in the scoring of levels of the learning curve, the curve's value could be improved for its utilization in similar learning environments.

The last figure shows the progression of learning scores (vertical axis) with increasing practice times (horizontal axis) via percentile lines, including 3%-97% and 15%-85% and 50%. The curved lines on the chart show selected percentiles that indicate the score rank. This curve is constantly going upwards, and it simply represents the average necessary practice times for any level of competency. It must be noted that if ABG sampling practices are 7 times, 97% (up to the 3% percentile line) of people reach 90-100 of skill scores, 70% (between 15% and 85% percentile lines) of them reach 95-100 of skill scores, 50% of people reach skill scores higher than 97, and less than 3% of people reach skill scores lower than 90.

It should be taken into account that the percentile ranking curve is an important model. It would allow the comparison of lower and higher percentile line rates. According to this curve, the percentile line changes faster with the primary higher score than the lower one and it reaches a score of 100 while the lower one finally reaches a score of 90 with 7 practices. By this diagram, it can be confidently said that with high and low prior skill levels, the nurses would obtain the minimum skill score of 90 with 7 practice times.

Utilization of this model in nurse training may have some advantages such as training standardization and its cost-effectiveness via repetition of practices in needed times, reducing iatrogenic damages of patients resulting from the excessive repetition of practices and upgrading the training quality of nursery students at any level of prior proficiency.

This scientific method is reusable and can be experienced in different educational environments and can help develop the practice level of training in the nursing field. It is suggested that the learning curve be taken into account in future studies in the standardization of other basic skill learning.

### 4.1. Strengths and Limitations

The strengths of the study were the steps of checklist design, the analysis model, and the results. The relaimpo package [22] provides various metrics to assess the relative importance in linear models, and it is a reference for comparison of how linear regression measures the variable importance. So, this measurement in the learning study increases the validity of the study. The findings of the study were shown in the way of reusable figures, and results would be easily applied to ABG sampling educational programs. This study had some limitations, including lack of a control group, random allocation, and gradual inclusion of participants.

## 5. Conclusion

Utilization of the learning curve could be helpful in the standardization of clinical practices in nursing education and the frequency of skill practice optimization, thus improving the education quality in this field. According to the learning curve, newly registered nurses in the ICU can reach an acceptable competency after 7 practices of ABG sampling. Also, the extent of newly registered nurses' prior competency can be a determining factor in the experience times needed for obtaining the specific level of proficiency.

## Figures and Tables

**Figure 1:** Study design for developing and testing a standardized learning curve for ABG sampling competency for nurses.

**Figure 2:** Box plot for scores for mastery in arterial blood gas.

**Figure 3:** Mean score for mastery in arterial blood gas (learning curve).

**Figure 4:** Mean change in score for mastery in arterial blood gas among times of experience.

**Figure 5:** Poisson model accuracy in predicting the number of times essential for mastery in arterial blood gas according to the cutoff point of the learning curve.

**Figure 6:** Distribution of time essential for mastery in arterial blood gas according to the cutoff point of the learning curve.

**Figure 7:** Percentile curve for scores for mastery in arterial blood gas. This graph presents the rate of increasing skill scores of nurses according to the number of practices. The black line indicated the median of scores, the red line indicated the percentile between 3 and 97%, and the green line indicated the percentile from 15% to 85%. The percentile from 3-15 is assumed the weak level, 15-50% is assumed the middle level, 50-85% is assumed a good level, and 85-90% is assumed a well level.

**Table 1:** Descriptive characteristics of newly registered nurses who participated in the ABG sampling competency study.

Variables		Frequency	Percentage
Sex	Male	19	33.9
	Female	37	66.1
Dominant hand	Right	50	89.3
	Left	6	10.7
Colleagues' cooperation	Very desirable	22	39.3
	Desirable	28	50.0
	Undesirable	6	10.7
Working shift	Morning working	13	23.2
	Evening working	14	25.0
	Night working	16	28.6
	Circulating working	13	23.2
Supervisor	Continuous	26	46.4
	Intermittent	28	50.0
	Sporadic	2	3.6

**Table 2:** Final checklist with three domains of the ABG sampling competency study.

Domains of the checklist		Importance coefficient
Before ABG sampling	Syringe heparinizing	3
	Checking heparin in the syringe	2
	Providing alcohol cotton	3
	Providing the pad under the patients' hand	2
	Informing the patient about the procedure	5

During ABG sampling	Correct nurse positioning	1
	Correct patient positioning	5
	Correct disinfection	5
	Relaxed the patient	5
	Taking the needle in the right way	4
	Entering the correct angle	4
	Appropriate management of the needle in an artery	4
	Getting the right amount of blood	2

After ABG sampling	Preventing patient from bleeding	5
	Correctly taping the puncture site	4
	Exporting air bubbles entering the needle	2
	Correct maintenance of blood samples	4
	Sending blood samples to the laboratory timely	3

**Table 3:** Estimates of relative importance (decomposed *R*^2^) of predictors for the linear regression model under the entering method in R software.

Covariate	Competency score time in arterial blood gas sampling						
	First	Second	Third	Fourth	Fifth	Sixth	Seventh
Age	0.018	0.005	0.003	0.013	0.003	0.007	0.013
Sex	0.081	0.032	0.018	0.016	0.005	0.005	0.003
Marriage	0.002	0.006	0.042	0.005	0.005	0.015	0.002
BMI	0.003	0.018	0.044	0.054	0.074	0.068	0.011
Major hand	0.071	0.037	0.026	0.052	0.058	0.081	0.019
GPA	0.006	0.014	0.011	0.009	0.006	0.018	0.011
Major satisfaction	0.066^∗^	0.101^∗∗^	0.070^∗^	0.047	0.079^∗^	0.035	0.046
Colleague's cooperation	0.011	0.018	0.017	0.009	0.008	0.004	0.005
Present supervisor	0.017	0.027	0.011	0.020	0.004	0.003	0.046
Shift	0.022	0.062	0.106	0.111	0.053	0.036	0.047
Preeducation	0.179^∗∗^	0.165^∗∗∗^	0.077^∗^	0.059^∗^	0.076^∗^	0.025	0.040
*R* ^2^	47.65%	48.73%	42.38%	39.67%	37.3%	29.93%	24.35%

^∗^0.05, ^∗∗^0.001, and ^∗∗∗^0.0001.

## Data Availability

Data are available from the first and corresponding authors upon reasonable request.

## References

[1] Hunsicker J., Chitwood T. (2018). High-stakes testing in nursing education: a review of the literature. *Nurse Educator*.

[2] Dobrowolska B., McGonagle I., Jackson C. (2015). Clinical practice models in nursing education: implication for students' mobility. *International Nursing Review*.

[3] Canzan F., Marognolli O., Bevilacqua A. (2017). An overview of clinical practice education models for nursing students: a literature review. *Assistenza infermieristica e ricerca*.

[4] Berndtsson I., Dahlborg E., Pennbrant S. (2020). Work-integrated learning as a pedagogical tool to integrate theory and practice in nursing education - an integrative literature review. *Nurse Education in Practice*.

[5] Lam C. K., Schubert C. (2019). Evidence-based practice competence in nursing students: an exploratory study with important implications for educators. *Worldviews on evidence-based nursing.*.

[6] Thomas C. M., Kellgren M. (2017). Benner's novice to expert model: an application for simulation facilitators. *Nursing Science Quarterly*.

[7] Belita E., Yost J., Squires J. E., Ganann R., Burnett T., Dobbins M. (2018). Measures assessing attributes of evidence-informed decision-making (EIDM) competence among nurses: a systematic review protocol. *Systematic Reviews*.

[8] Cinar F. I., Vesile Unver R., Seven M., Fidanci B. E., Cicek H. S., Yava A. (2014). Determination of the frequency of clinical skills implementation by senior nursing students in an emergency department. *International Journal of Caring Sciences*.

[9] Wallace M. W., Solano J. J. (2019). Radial Artery Cannulation. *StatPearls*.

[10] Chism L. A. (2017). *The Doctor of Nursing Practice*.

[11] Bailey C. D. (1989). Forgetting and the learning curve: a laboratory study. *Management Science*.

[12] Barrington M. J., Viero L. P., Kluger R., Clarke A. L., Ivanusic J. J., Wong D. M. (2016). Determining the learning curve for acquiring core sonographic skills for ultrasound-guided axillary brachial plexus block. *Regional Anesthesia and Pain Medicine*.

[13] Nguyen B. V., Prat G., Vincent J. L. (2014). Determination of the learning curve for ultrasound-guided jugular central venous catheter placement. *Intensive Care Medicine*.

[14] Speelman C. P., Kirsner K. (2005). *Beyond the Learning Curve: The Construction of Mind*.

[15] Lapré M. A., Nembhard I. M. (2011). Inside the Organizational Learning Curve: Understanding the Organizational Learning Process. *Foundations and Trends® in Technology, Information and Operations Management*.

[16] Pusic M. V., Boutis K., Pecaric M. R., Savenkov O., Beckstead J. W., Jaber M. Y. (2017). A primer on the statistical modelling of learning curves in health professions education. *Advances in Health Sciences Education: Theory and Practice*.

[17] Wang H. E., Seitz S. R., Hostler D., Yealy D. M. (2005). Defining the learning curve for paramedic student endotracheal intubation. *Prehospital Emergency Care*.

[18] Zhang X., Tanigawa N. (2009). Learning curve of laparoscopic surgery for gastric cancer, a laparoscopic distal gastrectomy-based analysis. *Surgical Endoscopy*.

[19] Prasad M. S. R., Manivannan M., Manoharan G., Chandramohan S. M. (2016). Objective assessment of laparoscopic force and psychomotor skills in a novel virtual reality-based haptic simulator. *Journal of Surgical Education*.

[20] Burke L. M. (2006). The process of integration of schools of nursing into higher education. *Nurse Education Today*.

[21] Jaber M. Y. (2016). *Learning Curves: Theory, Models, and Applications*.

[22] Grömping U. (2006). Relative importance for linear regression in R: the package relaimpo. *Journal of Statistical Software*.

[23] Lynch F. (2009). Arterial blood gas analysis: implications for nursing. *Nursing Children and Young People*.

[24] Grantcharov T. P., Bardram L., Funch-Jensen P., Rosenberg J. (2003). Learning curves and impact of previous operative experience on performance on a virtual reality simulator to test laparoscopic surgical skills. *American Journal of Surgery*.

[25] Loukas C., Nikiteas N., Kanakis M., Moutsatsos A., Leandros E., Georgiou E. (2010). A virtual reality simulation curriculum for intravenous cannulation training. *Academic Emergency Medicine*.

[26] Park I. J., Choi G. S., Lim K. H., Kang B. M., Jun S. H. (2009). Multidimensional analysis of the learning curve for laparoscopic colorectal surgery: lessons from 1,000 cases of laparoscopic colorectal surgery. *Surgical endoscopy*.

[27] Thomas R. C. (2012). *Long Term Human-Computer Interaction: An Exploratory Perspective*.

[28] Speelman C. P., Kirsner K. (2001). Predicting transfer from training performance. *Acta psychologica*.

[29] Ferguson E., James D., Madeley L. (2002). Factors associated with success in medical school: systematic review of the literature. *BMJ*.

[30] Lumb A. B., Vail A. (2004). Comparison of academic, application form and social factors in predicting early performance on the medical course. *Medical Education*.

